# Research on the Construction of College Students' Mental Health Security System

**DOI:** 10.1155/2022/4001603

**Published:** 2022-02-28

**Authors:** Hui Gao

**Affiliations:** Jilin Engineering Normal University, School of Education, Changchun 131400, China

## Abstract

With the development of modern society, people are increasingly pursuing quality of life and paying more attention to mental health education. Mental health education in colleges and universities should also conform to the development of the times, constantly reform the education mode, and help college students establish a healthy psychological environment, so as to better promote the growth of college students. From the perspective of positive psychology, a new idea of mental health education for college students has gradually emerged, that is, from the traditional negative intervention on college students' psychological problems to positive mental health education. Strengthening the mental health education of college students is an important measure to fully implement the Party's educational policy and implement quality education under the new situation, an important way and means to promote the all-round development of college students, and an important part of moral education in colleges and universities. College students' mental health education should be guided by the theory of positive psychology, start with family, society, school, and other aspects to build a brand-new mental health education guarantee system, and finally achieve the purpose of improving college students' psychological quality.

## 1. Introduction

Positive psychology studies discusses mental health problems from a positive perspective, which has become a new direction and mainstream of mental health research [1]. From the perspective of positive psychology, the new ideas of college students' mental health education are gradually emerging, that is, from the traditional negative intervention to the positive mental health education [2]. The curriculum system of college students' mental health education is the core content of college students' mental health education system, and it is an important link to carry out college students' mental health education [3]. How to pay attention to the organic combination of classroom teaching and extracurricular teaching in practice, carry out systematic education, and make full use of the advantages of various forms of education are important practical tasks and topics in front of college students' mental health educators. The development and rise of positive psychology not only provide a theoretical basis for college students' mental health education but also provides a practical basis for the construction of college students' mental health education curriculum system [4]. College students' mental health education should be guided by the theory of positive psychology, start from family, society, school, and other aspects, build a new mental health education security system, and ultimately achieve the purpose of improving college students' psychological quality [5].

Improving the security conditions is a necessary condition for the effective development of college students' mental health education. It is very important for colleges and universities to improve the security system of mental health education, better accept college students' mental health problems, and provide them with the opportunity to get help [6]. Attaching importance to the development of mental health education in colleges and universities and actively intervening in the psychology of college students are of great significance to the cultivation of talents in colleges and universities, the physical and mental health of college students and the harmonious development of the whole society [7]. Strengthening college students' mental health education is an important measure to comprehensively implement the party's education policy and quality education under the new situation, an important way and means to promote the all-round development of college students, and an important part of moral education in colleges and universities [8]. In practice, paying attention to the organic combination of classroom teaching and extracurricular teaching, carrying out systematic education, and making full use of the advantages of various forms of education are the important topics in the current college students' mental health education curriculum construction [9]. In the actual construction process, it should be based on the actual psychological characteristics of college students, using multimedia network technology, to build a systematic teaching platform for students' autonomous learning and communication.

## 2. The Problems of College Students' Mental Health Education Security System

### 2.1. The Guarantee System of Mental Health Education Lacks Operability

When carrying out mental health work in colleges and universities, the main target is the students in some psychological early warning database, while the psychological problems of the students outside the database are often ignored, lack of psychological disease prevention mechanism and developmental psychological education concept, which will limit the management effect of mental health and the popularity of mental health education. Influenced by traditional psychology, the mental health education of college students in China is mostly problem-oriented, and the course of mental health education of college students is no exception. The system of psychological crisis prevention is lack of standardization, and the implementation of the system is not in place. The reasons for the lack of operability of the mental health education security system are as follows: it started late, the development of related research is slow, the number of researchers is small, and a mature system has not yet been formed.

Colleges and universities need the guidance of correctly dealing with interpersonal relationships to guide students to correctly deal with all kinds of unfair phenomena, tolerate, let people, deal with things calmly, and treat people rationally. The cultivation of frustration tolerance and will can educate students to withstand setbacks and withstand blows. Students' steely will and tenacious struggle spirit has to be cultivated, so as not to be depressed by temporary setbacks. Education has to establish a correct outlook on job selection, etc.

The traditional mental health education curriculum for college students mainly focuses on the secondary goal, that is, problem-oriented. It pays more attention to the preventive goal of college students' mental health education and often ignores the developmental goal of college students' mental health education, that is, it lacks the development of college students' psychological potential and the cultivation of positive quality. Traditional psychology mainly focuses on the psychological problems or mental diseases of college students and ignores their psychological feelings. Positive psychology puts forward two concepts: prevention of mental illness and promotion of mental health. Positive psychologists believe that prevention is the method and measure to avoid the occurrence of problems or find the root of problems and reduce the extreme consequences caused by psychological problems [10]. Because of the convenience of its conditions, the richness of teachers, and the convenience of collecting samples, colleges and universities have obvious research advantages. Colleges and universities can provide research results needed by the society. However, in reality, colleges and universities often lack the research mechanism of mental health education guarantee and need to improve in providing honor, funding, and encouraging teachers to research related topics.

### 2.2. The Management System of Mental Health Organization Is Not Perfect

College students' mental health education course is different from other courses. Due to the particularity of people's psychological development, the course should pay more attention to college students' emotional experience and psychological experience in the teaching process. At present, most of the mental health education courses for college students are based on indoctrination education, and the classroom atmosphere is relatively dull. The single teaching method leads to the poor effect of the course. Of course, a large part of the reason is that there are many students choosing courses, and the teaching methods such as group counseling, situational experience, role play, and workshop cannot be effectively used. Due to the limited conditions, the files that college students set up when they enter the campus are not comprehensive enough, and the mental health files are not set up before they enter the school. It is necessary to scientifically build and manage the mental health files of college students and dynamically monitor the mental health status of college students. In the actual teaching process, some teachers have not been able to build a reasonable guarantee system for students' actual psychological problems. As a result, students lose interest in mental health education, and their psychological problems are becoming more and more serious.

As the future pillars of society, college students are in the key stage of self-awareness development. For example, only focusing on solving students' psychological problems or mental diseases cannot give full play to students' potential and promote the improvement of college students' psychological quality. College students have to be actively guided to feel the good time in life and experience the daily happy life in life. If college students have a substantial sense of happiness in life, they can extend this sense of happiness to the whole psychological state, hold a positive attitude to everything, and form a virtuous circle. Teachers still use a lot of academic language in the video process, which makes it difficult for students to understand the knowledge contained in it, and has a negative impact on students to create a healthy psychological environment. In the video teaching process, teachers ignore the use of body language, only relying on written language, it is difficult to reflect the key content of mental health education, and students can not enhance their interest in mental health learning. The highest goal of mental health education is to create a positive and healthy campus environment on campus. Through a good campus environment, college students can experience the fun of life in a positive environment and promote the healthy development of college students.

## 3. Countermeasures to Improve the Guarantee System of College Students' Mental Health Education

Psychological crisis intervention system is often needed in an emergency, so we cannot simply ignore its existence after it is published. Instead, it should be published on the common websites of colleges and universities and publicized among students' peers, which has achieved its effectiveness. The work of mental health education should strengthen the contact between the members of educational institutions and specific instructors, timely understand the work requirements of the members of the leading institutions, and also facilitate the support of school leaders at all levels for mental health education. Under the protection of national policies, college students' mental health education has experienced the development process from a difficult start to rapid popularization and has made remarkable achievements, but there are still some problems restricting their own development. The person in charge of the psychological center and the counselors in charge carry out the secondary management, take charge of the advisory service and teaching guidance work, and also play the role of administrative guidance and business guarantee in the management work. Other counselors and peer teams implement three-level management, which is responsible for paying attention to students' ideological and psychological dynamics, and providing guidance for related problems. It is obvious that the mental health education of college students is carried out in the school, while the environment that students are exposed to is composed of family, school, and society [11]. Therefore, the construction of college students' mental health education security system is inseparable from the positive efforts of family, school, and society [12].

The biggest advantage of effective research in school environment is that it is convenient to collect data from student samples. Compared with the experiment based on the laboratory, it is characterized by convenience and uniformity. As a result, samples obtained in the context of schools may have more ecological validity characteristics than those recruited in laboratory-based clinical trials.  Figure 1 shows the perception system architecture of mental health security system management.

The evaluation of personnel training is divided into six intervals, and the specific division is shown in Table 1. The relationship between normalized value and personnel training evaluation is shown in Figure 2.

Compared with academic courses, college students' mental health education pays more attention to students' current living conditions and emotional experiences. Therefore, elective courses mainly focus on psychological problems or psychological experiences that college students often encounter during their college years. According to positive psychology, when people live in society, they will have cognition of themselves, others, and various natural entities and their relations. Under the current social pressure, college students change from the student role to work role. Whether this stage can make a good transition and adapt to the society has a great influence on college students' mental health. In the complex campus environment, college students will encounter various problems in interpersonal communication. During the growth of each college student, they especially hope to have pleasant communication with others, intimate friends and classmates, and healthy interpersonal relationships after entering the university. Generally, colleges and universities have established psychological health records of college students, but they lack dynamic monitoring. After collecting students' related information and establishing mental health records, we should analyze and evaluate the situation that affects the development of students' mental health, combine the law of natural development, and integrate the common psychological problems in colleges and universities, which can predict the mental health of college students. In classroom teaching, we should actively guide students to change their perspectives and ways of looking at problems, face problems in life with a positive attitude, and face their own lives optimistically. Frustration will also become our driving force. The structure of the psychological prevention method based on college students' mental health security system is shown in Figure 3.

In the curriculum concept, we should take the positive concept as the guide and pay attention to the cultivation of the positive psychological quality of college students. The positive psychological quality of college students includes positive cognitive quality, emotional quality, will quality, moderate motivation system, good ability, and personality. Teachers can make students recall those successful experiences, feel the joy of success, and improve their self-esteem by meditation and self-experience in class. Students' mental health status is a dynamic process. No matter whether it is electronic files or paper files, it cannot only simply record the situation and find it when needed in the future but also play a role in preventing college students' psychological problems, screening out college students with potential mental health problems, giving them special counseling and intervening in psychological crisis. According to the three-level goal of college students' mental health education, the contents of college students' mental health education courses can be divided into developmental courses, preventive courses, and intervention courses. Among them, developmental courses pay attention to the shaping and training of positive emotions and positive personalities of college students, and the development of psychological potential and positive psychological quality of college students. A good campus culture environment can infiltrate healthy spirit into students, influence their behavior habits, create a good campus culture atmosphere, concentrate students' attention on campus culture, dilute their negative emotions caused by homesickness, academic problems, interpersonal problems, employment pressure and other reasons, cultivate their noble sentiments, and prevent the breeding of college students' bad psychological problems.

## 4. Conclusions

The guarantee system of college students' mental health education is highly professional and operational. With the frequent occurrence of college students' psychological problems, colleges and universities pay more and more attention to the construction of mental health education guarantee system and mental health education has made great progress than before. College students' mental health education is to enable students to know themselves deeply and to teach students positive quality training, life frustration education, life education, and so on through the reform of curriculum teaching and the improvement of curriculum content. As a new direction of psychological research, positive psychology's working goal reflects fraternity and humanity in the social sense, which is consistent with the goal of human development. Colleges and universities should increase the investment in mental health education, improve the existing equipment and facilities of mental health education and counseling centers and psychological counseling rooms, and build standardized individual and group counseling rooms and psychological catharsis, so as to create conditions for further developing individual and group psychological counseling. Colleges and universities actively respond to the call of the state and integrate mental health education into the teaching content to help college students form a healthy psychological environment so that college students can have a positive and good attitude in their future life and work.

## Figures and Tables

**Figure 1:** Perception system architecture.

**Figure 2:** The relationship between normalized value and talent training evaluation.

**Figure 3:** The structure of physical prevention methods.

**Table 1:** Classification of talent training evaluation.

Personnel training evaluation parameters	0–20	20–40	40–60	60–80	80–100
Normalized value	0.15	0.3	0.45	0.6	0.75

## Data Availability

The data used to support the findings of this study are included within the article.

## References

[1] Wu G. (2017). Research on the mental health education guarantee system of college students from the perspective of positive psychology. *Health Vocational Education*.

[2] Kang G. (2018). Analysis on the construction of the internal security system for college students’ labor rights and interests. *World of Labor and Social Security*.

[3] Acharya L., Jin L., Collins W. (2018). College life is stressful today–Emerging stressors and depressive symptoms in college students. *Journal of American College Health*.

[4] Liu K. (2016). Analysis on the construction of the secondary mental health education module system in colleges and departments. *NewWest*.

[5] Ji X., Xie J. (2015). The construction of college student’s mental health curriculum system from the perspective of general education. *Journal of Chifeng University (Nature Edition)*.

[6] Baloran E. T. (2020). Knowledge, attitudes, anxiety, and coping strategies of students during COVID-19 pandemic. *Journal of Loss and Trauma*.

[7] Zhao S. (2018). Research on the construction of mental health education system in higher vocational colleges from the perspective of sociology. *Journal of Science Education*.

[8] Zhou X. (2016). Research on the problems and countermeasures in the operation of the mental health service system for urban and rural residents. *Journal of Baoji University of Arts and Sciences*.

[9] Yu H., Xu X. (2019). Research on the psychological crisis and intervention system of college students in higher vocational colleges. *Journal of Hebei Tourism Vocational College*.

[10] Guo M., Lu J. (2020). Analysis on the causes and countermeasures of the mental health problems of vocational college students. *Chinese and Foreign Corporate Culture*.

[11] Zhuang M. (2019). Research on the mental health education innovation of university students from the perspective of big data. *Journal of Heilongjiang Vocational College of Ecological Engineering*.

[12] Chen Y. (2015). Prospects of mental health education for college students of science and technology. *Journal of Chifeng University (Nature Edition)*.

